RETRACTED

# Metoprolol Mitigates Ischemic Heart Remodeling and Fibrosis by Increasing the Expression of AKAP5 in Ischemic Heart

**DOI:** 10.1155/2022/5993459

**Published:** 2022-10-04

**Authors:** Feng Zhu, Qiushu Wang, Zhi Wang, Xu Zhang, Benkai Zhang, Hegui Wang

**Affiliations:** Department of Cardiology, Yijishan Hospital of Wannan Medical College, Wuhu, China

## Abstract

The harm of heart failure mainly causes patients to develop dyspnea, fatigue, fluid retention, and other symptoms, which impair patients' activity tolerance and lead to a dramatic decrease in patients' quality of life. The purpose of this study was to verify whether metoprolol regulates AKAP5 expression and test the role of AKAP5 postinjury in mitigating cardiac infarction-associated tissue remodeling and fibrosis. Sprague-Dawley (SD) rats underwent coronary artery ligation (CAL), which was followed immediately with metoprolol daily. And western blot and coimmunoprecipitation experiments were performed to detect the expression of related proteins in the sham-operated group, model group, and drug-treated group. HW/BW ratio and cardiac expression of COL1 and COL3 were increased in rats following CAL compared with shams. Treatment with metoprolol postinjury was associated with a decrease in HW/BW ratio and COL1/COL3 expression compared to uncontrolled rats. CAL resulted in decreased cardiac AKAP5 expression compared to the control group, while metoprolol treatment restored levels compared to baseline shams. Cardiac expression levels of NFATc3/p-NFATc3 and GATA4 were modest at baseline and increased with injury, whereas metoprolol suppressed gene expression to below injury-associated changes. Immunoprecipitation indicated that AKAP5 could bind and regulate PP2B. In summary, we know that metoprolol alleviates ischemic cardiac remodeling and fibrosis, and the mechanism of alleviating remodeling may improve cardiac AKAP5 expression and AKAP5-PP2B interaction.

## 1. Introduction

Patients with heart failure have severely diminished systolic as well as diastolic function and diminished cardiac pumping. Heart failure (HF) has many hazards that can affect the quality of life, affect organ function, and be life-threatening. Recent results from epidemiological surveys of HF in China show a weighted HF prevalence of 1.3%, or approximately 13.7 million HF patients, among our population of residents aged ≥35 years. The incidence of HF continues to rise as the population ages [1, 2]. Unfortunately, HF is minimally symptomatic even with real cardiac structural changes such as left ventricular (LV) hypertrophy, LV systolic or diastolic dysfunction, and valvular disease. The prognosis for advanced HF is poor. Therefore, early intervention is likely to be more impactful in reducing morbidity and mortality.

RETRACTED

LV remodeling (LVR) is common after ischemic myocardial injury and manifests as changes in ventricular thickness and size. This compensation mechanism initially minimizes cardiac dysfunction but, over time, proves inadequate at maintaining cardiac function [3]. Postischemic cardiac remodeling is worsened by chronic activation of the neuroendocrine system and unrestrained extracellular matrix deposition. Several cytokines and hormones promote this process, including hyperactive beta-adrenocortical hormones, and are found to increase in animal models and people with cardiac remodeling [4]. Ventricular remodeling is caused by a complex series of cellular and molecular mechanisms leading to progressive changes in ventricular weight, volume, and morphology of cardiomyocytes and the myocardial matrix, characterized by progressive dilation of the primary Mi region and LV volume. It begins in the early stage of AMI and is a response of the myocardium to myocardial injury and cardiac overload. Recent studies have shown that changes in the structure and composition of the extracellular matrix of cardiac muscle are an early event in the progression of left ventricular myocardial remodeling and cardiac pump dysfunction and have an important role in myocardial remodeling [5].

Chronic heart failure is a slow process, often taking over a decade for symptoms to develop. In this process, the heart is engaged in a constant interplay with the organism, with the impact of the neuroendocrine system being most pronounced. This is mainly manifested in the remodeling of the myocardium. Any single organ and tissue of an organism have a certain structure-activity relationship, and what structure determines what function it performs. In turn, because an organism requires such a function, an organ or tissue evolves progressively into its present-day shape. Thus, an organ lesion, although not necessarily one in which a structural change occurs, must illustrate that the organ has developed the lesion. Structural alterations are accumulated in response to a variety of humoral and cellular factors as well as various receptors for prolonged periods [6]. For myocardial remodeling, because the myocardium is nonrenewable, hypertrophy, apoptosis, and remodeling of the glial network outside the cardiomyocyte can be used as entry points to explain myocardial remodeling. In the RAS system, *β* Adrenergic system, the role of the sympathetic system in promoting ventricular remodeling has been demonstrated several times. The ECM plays an important role in maintaining the structural and functional integrity of the heart, and disruption of the dynamic balance between myocardial interstitial fibrillar collagen synthesis and degradation damages the microenvironment of the heart, which has also been confirmed to be associated with the ventricular remodeling in recent years and is gaining increasing attention [7].

RETRACTED

AKAP5, also known as akap79/150, includes a variety of proteins of different genera encoded by the homologous gene AKAP5, including bovine akap75, human akap79, and rat and mouse AKAP150 [8]. Under normal physiological conditions, akap79/150 can affect cardiac myocytes. The signal transduction and sensitize recycling of adrenaline receptors [9], regulation of the cardiac hypertrophy signal [10], and the coupling of excitation-contraction, relaxation, and intracellular calcium circulation [10–12] in cardiac cells are involved in ensuring the normal function and morphology of the heart. In arrhythmia, AKAP150 acts in two ways: it intensifies arrhythmia caused by calcium channel-related gene mutation [13], and it may have a therapeutic effect on arrhythmia caused by potassium channel-related gene mutation [14, 15].

*β*1-adrenergic receptor (*β*-AR) stimulation *in vitro* and *in vivo* increased the expression and activity of matrix metalloproteinases 2 and 9 (MMP-2 and MMP-9) in cardiac myocytes [16]; it also induced cardiomyocyte apoptosis [7, 17, 18]. In addition, *β*1-AR–mediated increase in cyclic adenosine monophosphate was greater in AKAP5 null myocytes [19]. There are few studies on the role of AKAP5 in cardiac function, especially there are few studies on the role of AKAP5 to regulate myocardial remodeling and fibrosis after myocardial infarction. The focus of this article is on whether *β*-AR blockers regulate the expression of AKAP5 and the downstream signal protein after myocardial infarction.

However, how or if AKAP5 participates in the regulation of *β*1-ARs in ischemic cardiac remodeling is minimally studied. Herein, we tested the hypothesis that therapy with selective *β*1-AR blocker metoprolol can ameliorate ischemic cardiac remodeling by alerting AKAP5 levels.

## 2. Materials and Methods

### 2.1. Animals

Adult male Sprague-Dawley (SD) rats (~200 g/animal) were obtained from the Zhejiang Experimental Animal Center of Zhejiang University (Hangzhou, China; License No. [SCXK (Zhen) 20140001]). The animals were raised in the Central Laboratory Animal Room of the Rocky Mountain Hospital of Wannan Medical College (Wuhu, China). All animal experimental protocols used in this study were approved by the Ethics Committee of Yanjishan Hospital of Wannan Medical College and met the guidelines for the use of live animals.

### 2.2. Reagents and Equipment

Bicinchoninic Acid (BCA) protein quantification kits were from the Bey time Institute of Biotechnology (Nanjing, China). Antibodies to AKAP5, NFATc3, p-NFATc3, and GATA4 were from Santa Cruz Biotechnology (Dallas, Texas, US). Antibody to PP2B was from Cell Signaling Technology (CST; Beverly, Massachusetts, US), and COL1 and COL3 were from Abcam (Cambridge, UK). The chemiluminescence imager was from Tanon Science & Technology Co., Ltd. (Shanghai, China), and the microplate reader was from Bio-Rad Laboratories, Inc. (Hercules, California, US).

RETRACTED

### 2.3. Myocardial Infarction Model

50 adult male Sprague-Dawley (SD) rats were anesthetized by intraperitoneal injection of 10% chloral hydrate (0.3 mL/100 g) and connected to an RM6240 Multi-path Physio meter (Chengdu Instrument Factory, Chengdu, China). After tracheal intubation, animals were mechanically ventilated (Beijing Zhoushan Electronic Technology Co., Ltd., Beijing, China). Using sterile techniques, the thoracic cavity was opened between the third and fourth ribs on the left margin of the sternum, and a ligature was placed on the root of the left anterior descending coronary artery. Wounds were closed in layers. Sham animals underwent all procedures except coronary ligature. Animals were observed until fully recovered. Finally, five rats survived in each group. Of note, the rats should be housed in a single cage after surgery. Although rats themselves have a relatively strong anti-infection ability, prevention of infection is beneficial to promote postoperative recovery, and good postoperative care can improve the survival rate of animal models. Therefore, all surgical instruments used preoperatively were sterilized by 75% alcohol immersion. After surgery, 800000 U of penicillin was injected intraperitoneally. After the rat is anesthetized and awake, it is associated with sugar water and feeding without fasting. An appropriate amount of energy supplementation is available postoperatively. Winter should pay attention to education.

### 2.4. Study Design

The study groups with interventions were as follows. Overall, 50 rats were randomly divided into three groups for follow-up experiments, (1) a sham-operated control group (sham group) fed normal rat chow; (2) an injury group that underwent coronary artery ligation; (3) the third group was the metoprolol treatment group. The rats were treated with metoprolol (20 mg/kg/d) for 8 weeks. The sham and model groups were garaged the same amount of saline vehicle for 8 weeks. The rats were given intraperitoneal injections of appropriate amounts of pentobarbital sodium for sedation and analgesia for three consecutive days after the operation. The rats were euthanized by intravenous injection of 100 mg/kg of phenobarbital.

RETRACTED

### 2.5. Western Blot

On study completion, animals were humanely euthanized, and their hearts were excised. Tissue was homogenized in lysis buffer, agitated on wet ice for 30 mins, centrifuged at 12000 rpm, and then the supernatant was reserved. Measurement of total protein concentration was conducted using the BCA method. To detect protein concentration, we performed gel electrophoresis by loading equivalent amounts of protein in each group. After protein transfer, blots were incubated in bovine serum albumin at room temperature for 2 h. Following PBS washing, the corresponding primary antibodies (dilution, 1: 1000; Cell Signaling Technology, Inc., Danvers, MA, USA) were added and kept at 4°C for 14 h. After washing, blots were incubated with the secondary antibody at room temperature for 1 h, washed, and exposed to a chemiluminescence agent. ImageJ software (National Institutes of Health, Bethesda, Maryland, US) was employed to quantitate protein band expression.

### 2.6. Coimmunoprecipitation

The cardiac lysate was incubated with AKAP5 antibody (dilution, 1: 1000; Cell Signaling Technology, Inc., Danvers, MA, USA) or rabbit antimouse immunoglobulin G (1 : 3,000, Abcam, Cambridge, MA, USA) and incubated at 4°C for 14 h. Protein A/G agarose beads were added to the mixtures and incubated at 4°C for 4 h followed by centrifugation at 3000 rpm for 3 min. The supernatant was discarded, and beads were washed and boiled in water for 5 min. Samples were then subjected to western blot as detailed above.

### 2.7. Statistical Analysis

SPSS version 18.0 was used for statistical analysis. Statistical differences among groups were assessed using a two-tailed Student's *t*-test (two experimental groups) or ANOVA (three or more groups). *p* < 0.05 was considered statistically significant. The results have expressed the means ± SD, n ≥ 3.

## 3. Results

### 3.1. Characterization of the Ischemic Cardiac Model

Gross observation found that before coronary ligature, hearts appeared bright red in color, and electrocardiogram waveforms were normal, as shown in Figure 1(a). After ligature, blanching of the cardiac wall was observed in the distribution of the left anterior descending coronary. Marked changes were also seen in the ECG. Specifically, the J point of lead II and the ST-T segment were uniformly elevated, as shown in Figure 1(b). These later results are consistent with ischemic myocardial infarction.

### 3.2. Ischemia-Mediated Increase in Cardiac Weight Is Ameliorated by Metoprolol

The ratios of heart weight to body weight (HW/BW) were determined by weighing heart samples from each group of rats and comparing them with the weight of the rats before sacrifice. Coronary ligation resulted in a significant increase in HW/BW ratio; this was attenuated in animals treated with metoprolol (*P* < 0.05, *n* = 5), as shown in Figure 2.

RETRACTED

### 3.3. Metoprolol Attenuates Matrix Protein Expression in Ischemic Hearts

Protein expression levels of matric genes COL1 and COL3 were greater in ischemia hearts compared to sham hearts. Metoprolol treatment was associated with a decrease in matrix protein expression in ischemic hearts (*P* < 0.05, *n* = 5), as shown in Figure 3.

### 3.4. Metoprolol Corrects Ischemia-Driven Changes in Cardiac AKAP5, P-NFATc3/NFATc3 and GATA4

Ischemia was associated with a decrease in cardiac AKAP5 compared to sham, which was attenuated by metoprolol attenuated (*P* < 0.05, *n* = 5), as shown in Figure 4(a) and Figure 4(b). In contrast, ischemia was associated with decreased cardiac p-NFATc3/NFATc3 and increased GATA4 compared to sham, and metoprolol suppressed these changes (*P* < 0.05, *n* = 5), as shown in Figure 4(c) to Figure 4(f).

### 3.5. Cardiac AKAP5 and PP2B Immunoprecipitated in Heart Tissue

Adrenergic receptors control cardiac function and size. In turn, AKAPs, and specifically AKAP5, regulate *β*-AR activity. PP2B is widely expressed in the heart and elsewhere and is reported to be complex with various AKAPs [20]. Consistent with this, AKAP5 and PP2B were colocalized by immunoprecipitation in cardiac samples, and this relationship appeared to change under ischemia and metoprolol treatment, as shown in Figure 5(a). Western blots of protein levels were found in samples employed in AKAP5, as shown in Figure 5(b).

## 4. Discussion

In preclinical models, heart injury and subsequent cardiac remodeling are commonly induced models via several techniques such as aortic-arch constriction [21], ischemia [22], toxic agents [23], and hypertension. Ischemic cardiac remodeling is characterized by organ hypertrophy, fibrosis, and functional deterioration [24]. Ischemic cardiac hemodynamic changes can induce heart failure via systolic dysfunction [25]. This process is potentiated by reflex sympathetic-nerve activation and the release of catecholamines such as norepinephrine and epinephrine [26]. While initially supporting ventricular contractility and heart rate to maintain cardiac output [27] long-term sympathetic-nerve activation is detrimental [28, 29]. The pathological mechanisms involved in creating animal models of congestive heart failure include pressure overload, volume overload, and decreased cardiac contractility. Myocardial ischemia causes a reduction in the number of cardiomyocytes and a decrease in cardiac contractility, and animal models are mainly used for experimental studies of pathophysiological changes and novel therapeutic approaches after myocardial ischemia. Many kinds of animals can be used for model making, easy to operate and observe, but they are expensive, so many researchers prefer to choose individual rats which are moderate and relatively inexpensive, and Sprague-Dawley rats and Wistar rats, which are a common choice. Coronary artery ligation and liquid nitrogen freezing of the left ventricle are commonly used methods in animal models of rats, and both can cause ischemia and necrosis of the left ventricular myocardium, and the former is mainly through stenosis or occlusion of the coronary artery to cause myocardial ischemia and infarction, and to cause heart failure by decreasing myocardial contractility; the greatest advantage is clinical relevance, but it is affected by many factors; the area of the infarct area is not easy to control, and the location often changes. The variation between animal models is large, and assays of cardiac function are prone to variability; However, the location of scar tissue caused by infarction in the frostbite model is relatively fixed, and the area size of the scar is also relatively constant, with little animal variation when cardiac function is measured, but with poor clinical relevance. The former was chosen given the advantages and disadvantages of each of the two models, and our experimental study design of stem cell transgenic therapy for CHD focused on maximizing clinical simulation.

RETRACTED

Metoprolol belongs to class 2A, that is, partially activated *β* 1-receptor blockers, which can slow down the rate of atrioventricular conduction, inhibit muscle contraction, and reduce dirty rhythmicity. After taking metoprolol, the drug was evenly dispersed in the gastrointestinal tract, and the drug was released steadily and steadily, which made the drug concentration stable, the peak concentration lower, and reduced the adverse reactions to the drug. And for patients with chronic “insufficiency” combined with muscle infarction, improve the visceral function of patients, reduce the incidence of abnormal incidence, reduce the death of patients, and reduce the pain of patients with chronic “insufficiency” combined with muscle infarction.

Herein, we established a model of acute cardiac ischemia and tested the role of the adrenergic blockade to revert the morphologic and gene-associated changes. The present study demonstrates, for the first time, that metoprolol can restore cardiac expression levels of AKAP5 and suppress the levels of p-NFATc3/NFATc3 and GATA4 and enhance cardiac AKAP5 and PP2B protein-protein interaction in rat chronic myocardial infarction model. The results indicate that treatment with metoprolol mitigates ischemic cardiac remodeling and fibrosis, which mechanism of mitigating remodeling likely to improve cardiac AKAP5 expression and AKAP5-PP2B interaction. Metoprolol can be a selectively antagonized *β*-1-adrenoceptor. Studies have shown that metoprolol can reduce the level of proinflammatory cytokine TNF-*α* and IL-1 [30, 31]. Similarly, metoprolol has a positive therapeutic effect on MI rats by inhibiting the expression of proto-oncogene protein [32, 33]. That is, *β* adrenergic blockade was tested against established cardiac changes. While the loss of adrenergic support may alter function to some degree, in this study, we found this treatment reverted or limited adverse cardiac remodeling and fibrosis. At the same time, changes in key genes involved in adrenergic signaling were improved. This included reversion of ischemia-mediated changes in cardiac AKAP5, p-NFATc3, and GATA4. Therefore, *β* adrenergic blockade may alter the interaction between AKAP5 and the general dephosphorylating enzyme PP2B (calcineurin). PP2B also altered NFAT activity [34] and is implicated in cardiac remodeling. Ventricular remodeling after myocardial infarction mainly includes hypertrophy and fibrosis of myocardial cells. The representative proteins of fibrosis are COL-1 and COL-3. In the experiment, protein expression of COL-1 and COL-3 was detected in the hearts of three groups of mice. COL-1 and COL-3 were significantly higher than in the control, and COL-1 and COL-3 were significantly higher than in the model group, indicating that metoprolol can slow myocardial fibrosis [35–37].

RETRACTED

This study has several limitations. First, the characterization of the ischemic model was morphologic and not correlated with functional outcomes. It would be useful to have also determined systolic and diastolic contractility, chamber volume, and cardiac output. Second, changes in gene protein levels do not equate with protein function. It will be useful to assess if target proteins had altered activity under the conditions of the model. Third, immunoprecipitation, while showing adherence, does not represent true molecular binding. Such interactions are further supported by advanced fluorescent microscopy.

In summary, the present study revealed that adrenergic blockade can resolve established ischemic cardiac remodeling and alter protein levels of key signaling intermediates, which mechanism of mitigating remodeling is likely to improve cardiac AKAP5 expression and AKAP5-PP2B interaction. Further research is needed to determine how and to what extent AKAP5 targets cardiomyocyte remodeling in the context of HF.

RETRACTED

## Figures and Tables

**Figure 1:** Ligation of the anterior descending coronary induces ischemia. Whole heart images showing heart color and ECG tracings before (a) and after myocardial infarction (b). Representative hearts and tracing are shown from a total of four animals.

**Figure 2:** Ischemia-mediated increase in cardiac weight is ameliorated by metoprolol. Rats were subject to ischemia ± metoprolol, and HW/BW ratios were determined. (a) Morphologic appearance of rat hearts in each group. (b) Calculated HW/BW ratios in each group of rats. ^∗^*P* < 0.05 indicates comparison with the sham group; ^#^*P* < 0.05 indicates comparison with the metoprolol-treated group.

**Figure 3:** Metoprolol attenuates matrix protein expression in ischemic hearts. Changes in expression levels of COL1 and COL3 proteins. (a and c) Western blot expression of COL1 and COL3 and respective densitometry. (b and d) ^∗^*P* < 0.05 indicates comparison with the sham group; ^#^*P* < 0.05 indicates comparison with the metoprolol-treated group.

**Figure 4:** Metoprolol corrects ischemia-driven changes in cardiac AKAP5, NFATc3, and GATA4 changes in AKAP5, NFATc3, and GATA4 expression during myocardial remodeling. (a, c, and e) Protein expression of AKAP5, NFATc3, and GATA4 was detected by western blot. (b, d, and f) Densitometry analysis of respective blots. ^∗∗^*P* < 0.01 indicates comparison with the sham group; ^#^*P* < 0.05 indicates comparison with the metoprolol-treated group.

**Figure 5:** Cardiac AKAP5 and PP2B immunoprecipitated in heart tissue. Immunoprecipitation pulldown displaying association of AKAP5 and PP2B. (a) In the AKAP5 coimmunoprecipitation experiment, the PP2B band was not noted in IgG control incubated samples. (b) Western blot showing the expression of AKAP5 and PP2B in samples employed in the coimmunoprecipitation experiment. AKAP5 was found to bind and regulate PP2B. ^∗^*P* < 0.05 indicates comparison to the sham group; ^#^*P* < 0.05 indicates comparison to the metoprolol-treated group.

## Data Availability

The simulation experiment data used to support the findings of this study are available from the corresponding author upon request.

## References

[1] Piepoli M. F., Adamo M., Barison A. (2022). Preventing heart failure: a position paper of the heart failure association in collaboration with the European Association of Preventive Cardiology. *European Journal of Preventive Cardiology*.

[2] Savarese G., Lund L. H. (2017). Global public health burden of heart failure. *Cardiac Failure Review*.

[3] Hotta V. T., Rassi D. D. C., Pena J. L. B. (2022). Critical analysis and limitations of the diagnosis of heart failure with preserved ejection fraction (HFpEF). *Arquivos Brasileiros de Cardiologia*.

RETRACTED

[4] Gautam S. (2022). Post-myocardial Infarction heart failure: a review on management of drug therapies. *Cureus*.

[5] Wang G., Liu X., Guo Z. (2022). Effect of entresto on clinical symptoms, ventricular remodeling, rehabilitation, and hospitalization rate in patients with both acute myocardial infarction and acute heart failure. *Evidence-based Complementary and Alternative Medicine*.

[6] Kwon J. S., Barr E. W., Chuprun J. K., Koch W. J. (2021). In Vivo Stimulation of *α*- and *β*-Adrenoceptors in Mice Differentially Alters Small RNA Content of Circulating Extracellular Vesicles. *Cells*.

[7] Singh K., Xiao L., Remondino A., Sawyer D. B., Colucci W. S. (2001). Adrenergic regulation of cardiac myocyte apoptosis. *Journal of Cellular Physiology*.

[8] Diviani D., Reggi E., Arambasic M., Caso S., Maric D. (2016). Emerging roles of A-kinase anchoring proteins in cardiovascular pathophysiology. *Biochimica et Biophysica Acta*.

[9] Nooh M. M., Mancarella S., Bahouth S. W. (2018). Novel paradigms governing *β*_1_-Adrenergic receptor trafficking in primary adult rat cardiac myocytes. *Molecular Pharmacology*.

[10] Li X., Matta S. M., Sullivan R. D., Bahouth S. W. (2014). Carvedilol reverses cardiac insufficiency in AKAP5 knockout mice by normalizing the activities of calcineurin and CaMKII. *Cardiovascular Research*.

[11] Nichols C. B., Rossow C. F., Navedo M. F. (2010). Sympathetic stimulation of adult cardiomyocytes requires association of AKAP5 with a subpopulation of L-type calcium channels. *Circulation Research*.

[12] Li L., Li J., Drum B. M. (2017). Loss of AKAP150 promotes pathological remodelling and heart failure propensity by disrupting calcium cycling and contractile reserve. *Cardiovascular Research*.

[13] Cheng E. P., Yuan C., Navedo M. F. (2011). Restoration of normal L-type Ca2+ channel function during Timothy syndrome by ablation of an anchoring protein. *Circulation Research*.

[14] Byrne D. P., Omar M. H., Kennedy E. J., Eyers P. A., Scott J. D. (2022). Biochemical analysis of AKAP-anchored PKA signaling complexes. *Methods in Molecular Biology*.

[15] Huang T., Zhang B., Wang Z., Wang Y., Li W., Wang H. (2020). AKAP5 anchors PKA to enhance regulation of the HERG channel. *The International Journal of Biochemistry & Cell Biology*.

[16] Krishnamurthy P., Subramanian V., Singh M., Singh K. (2007). *β*1 integrins modulate beta-adrenergic receptor-stimulated cardiac myocyte apoptosis and myocardial remodeling. *Hypertension*.

[17] Kumari R., Ray A. G., Mukherjee D., Kar D., Konar A., Bandyopadhyay A. (2022). Downregulation of PTEN Promotes autophagy via concurrent reduction in apoptosis in cardiac hypertrophy in PPAR *α*−/− mice. *Frontiers in Cardiovascular Medicine*.

RETRACTED

[18] Shizukuda Y., Buttrick P. M., Geenen D. L., Borczuk A. C., Kitsis R. N., Sonnenblick E. H. (1998). Beta-adrenergic stimulation causes cardiocyte apoptosis: influence of tachycardia and hypertrophy. *The American Journal of Physiology*.

[19] Li X., Nooh M. M., Bahouth S. W. (2013). Role of AKAP79/150 protein in *β*_1_-adrenergic receptor trafficking and signaling in mammalian cells. *The Journal of Biological Chemistry*.

[20] Li J., Aponte Paris S., Thakur H., Kapiloff M. S., Dodge-Kafka K. L. (2019). Muscle A-kinase-anchoring protein-*β*-bound calcineurin toggles active and repressive transcriptional complexes of myocyte enhancer factor 2D. *The Journal of Biological Chemistry*.

[21] Thum T., Gross C., Fiedler J. (2008). MicroRNA-21 contributes to myocardial disease by stimulating MAP kinase signalling in fibroblasts. *Nature*.

[22] Zhang Y., Köhler K., Xu J. (2011). Inhibition of p53 after acute myocardial infarction: reduction of apoptosis is counteracted by disturbed scar formation and cardiac rupture. *Journal of Molecular and Cellular Cardiology*.

[23] Potočnik N., Perše M., Cerar A., Injac R., Finderle Ž. (2017). Cardiac autonomic modulation induced by doxorubicin in a rodent model of colorectal cancer and the influence of fullerenol pretreatment. *PLoS One*.

[24] Heusch G., Libby P., Gersh B. (2014). Cardiovascular remodelling in coronary artery disease and heart failure. *The Lancet*.

[25] McKay R. G., Pfeffer M. A., Pasternak R. C. (1986). Left ventricular remodeling after myocardial infarction: a corollary to infarct expansion. *Circulation*.

[26] Mueller H. S., Ayres S. M. (1980). Propranolol decreases sympathetic nervous activity reflected by plasma catecholamines during evolution of myocardial infarction in man. *The Journal of Clinical Investigation*.

[27] Bhargava V., Shabetai R., Mathiäsen R. A., Dalton N., Hunter J. J., Ross J. (1998). Loss of adrenergic control of the force-frequency relation in heart failure secondary to idiopathic or ischemic cardiomyopathy ^1^. *The American Journal of Cardiology*.

[28] Benedict C. R., Johnstone D. E., Weiner D. H. (1994). Relation of neurohumoral activation to clinical variables and degree of ventricular dysfunction: a report from the registry of studies of left ventricular dysfunction. *Journal of the American College of Cardiology*.

[29] Omland T., Aarsland T., Aakvaag A., Lie R. T., Dickstein K. (1993). Prognostic value of plasma atrial natriuretic factor, norepinephrine and epinephrine in acute myocardial infarction. *The American Journal of Cardiology*.

RETRACTED

[30] Ahmed A. (2003). Myocardial beta-1 adrenoceptor down-regulation in aging and heart failure: implications for beta-blocker use in older adults with heart failure. *European Journal of Heart Failure*.

[31] Lu Y., Li L., Zhao X., Huang W., Wen W. (2011). Beta blocker metoprolol protects against contractile dysfunction in rats after coronary microembolization by regulating expression of myocardial inflammatory cytokines. *Life Sciences*.

[32] Grassi G. (2018). Metoprolol in the treatment of cardiovascular disease: a critical reappraisal. *Current Medical Research and Opinion*.

[33] Zhang S., Zhang M., Goldstein S. (2013). The effect of c-fos on acute myocardial infarction and the significance of metoprolol intervention in a rat model. *Cell Biochemistry and Biophysics*.

[34] Nie B., Liu C., Bai X. (2018). AKAP150 involved in paclitaxel-induced neuropathic pain via inhibiting CN/NFAT2 pathway and downregulating IL-4. *Brain, Behavior, and Immunity*.

[35] Prabhu S. D., Frangogiannis N. G. (2016). The biological basis for cardiac repair after myocardial infarction: from inflammation to fibrosis. *Circulation Research*.

[36] Li X., Xiang N., Wang Z. (2020). Ginsenoside Rg2 attenuates myocardial fibrosis and improves cardiac function after myocardial infarction via AKT signaling pathway. *Bioscience, Biotechnology, and Biochemistry*.

[37] Gyöngyösi M., Winkler J., Ramos I. (2017). Myocardial fibrosis: biomedical research from bench to bedside. *European Journal of Heart Failure*.

